The article "Breast diseases histologically diagnosed at a tertiary facility in Uganda (2005–2014)" was published in 2018. Journal: BMC Cancer.

# Breast diseases histologically diagnosed at a tertiary facility in Uganda (2005–2014)

**DOI:** 10.1186/s12885-018-5208-6

**Published:** 2018-12-22

**Authors:** Salvatore Ssemmanda, Eric Katagirya, Phiona Bukirwa, David Alele, Robert Lukande, Samuel Kalungi

**Affiliations:** 1 School of Medicine, Makerere University College of Health Sciences, Kampala, Uganda; 2 Department of Immunology and Molecular Biology, Makerere University College of Health Sciences, Kampala, Uganda; 3 Department of Pathology, Makerere University College of Health Sciences, Kampala, Uganda

## Abstract

**Background:**

The prevalence and distribution of histologically diagnosed breast disease are not well documented in low income countries, Uganda inclusive. Although the greater majority of breast lesions globally are benign, breast cancer is the most frequently diagnosed cancer all over the world. We aimed at documenting the prevalence of different breast diseases histologically diagnosed at the histopathology laboratory of the Department of Pathology of the Makerere University College of Health Sciences (MakCHS Lab) over a decade (2005–2014). We also describe the demographic characteristics of the patients in Uganda diagnosed with breast disease at the MakCHS Lab during the same period.

**Methods:**

This was a 10 year retrospective study of histologically diagnosed breast disease between 2005 and 2014 inclusive at the MakCHS Lab. We extracted information from hard copies of all 2510 histopathology reports retrieved from archives of the Department of Pathology at the MakCHS Lab. 640 records that were either damaged beyond recognition of key details, were duplicated, were implausible or had no conclusive diagnosis made were excluded. Information to be analyzed was then entered into Epidata (version 3.1) on a password protected laptop. Data analysis was done using SPSS software (v16 for Windows × 64).

**Results:**

From the 1870 patients’ records eventually analyzed, breast disease was most diagnosed in female patients (97.1%). The overall mean age for breast disease diagnosis was 33 years (S.D ± 16.46) and median age 26 years (IQR: 20–43). Fibroadenoma (40.1%) was the most diagnosed breast disease overall. We noticed steadily increasing frequency of diagnosis of cancerous breast diseases over the last half of the study period. Invasive ductal carcinoma was the most diagnosed breast cancer (326 cases, 55.6%). A high female to male breast cancer ratio of 48:1 was observed. The highest regional breast cancer proportion was from the Western region of the Country.

**Conclusions:**

There is need for more research into the picture of breast disease in the country, covering various demographic characteristics of the country’s population for all regions and informing about its incidence rates and prevalence and also the breast cancer risk estimate for benign breast disease.

The article "Breast diseases histologically diagnosed at a tertiary facility in Uganda (2005–2014)" was published in 2018. Journal: BMC Cancer.

## Background

Breast cancer is the most frequently diagnosed cancer in women all over the world [1]. Globally, nearly 1.7 million new cases of breast cancer were diagnosed in 2012, accounting for 25% of all cancer cases in women [2]. Amongst women from Sub-Saharan Africa however, it is second most frequent after cervical cancer [3]. Nonetheless, the greater majority of breast lesions globally are benign [4].

The prevalence of the different breast diseases is not well documented in low-income countries, Uganda inclusive. The scarcity of published data about these diseases means that little is known about the trends in the prevalence and incidence of the different breast diseases in these countries. Furthermore, little information is known about the demographic distribution of these breast diseases in these countries.

This study aimed at documenting the prevalence of different breast diseases diagnosed histologically at MakCHS Lab over a decade (2005–2014) by reviewing the laboratory diagnostic reports for all breast diseases during the said period. Further attempts were made at describing the demographic characteristics of the patients in Uganda diagnosed with breast disease at the laboratory. The study also describes the demographic characteristics of the patients in the country diagnosed with breast disease at the laboratory over the said study period.

## Methods

Hard copies of the laboratory histology reports were retrieved from the Department of Pathology archives for the years 2005 to 2014. Reports with samples identified as being from the breast were manually identified and grouped together by year. Information important for the study was then entered into Epidata (version 3.1) on a password protected laptop. The information transcribed included the age, sex, ethnicity, year of diagnosis and histological diagnosis made. During entry care was taken to ensure that only reports of breast disease were entered.

The data was saved in excel (.xls) and SPSS (.sav) formats. Data analysis was done using SPSS software (v16 for Windows × 64).

### Study site

The study was done at the Histopathology laboratory of the Department of Pathology at the Makerere University College of Health Sciences (MakCHS). It is located at the Mulago National Referral and Teaching Hospital in Kampala, Uganda. The laboratory is arguably the busiest histopathology laboratory in the country as it is the main public laboratory, serving the biggest hospital in the country and by far has the highest number of pathologists.

The article "Breast diseases histologically diagnosed at a tertiary facility in Uganda (2005–2014)" was published in 2018. Journal: BMC Cancer.

### Inclusion and exclusion criteria

All 2510 histopathology reports with breast disease diagnoses from primarily breast tissue samples made at the MakCHS Lab for the years 2005–2014 were included. 555 records that were damaged beyond recognition of key details or duplicated reports were excluded. This was followed by the exclusion of another 85 found implausible or noted to bear no conclusive diagnosis when the data entries were re-examined. The 85 records included 72 cases that were concluded as “no cancer tissue seen”. These were excluded to avoid diagnostic ambiguity as these could not be categorized pre-cancerous or otherwise benign. However the cases specified as “breast malignancy (18 cases)” or “adenocarcinomas (186 cases)” were included for analysis as these were evidently malignant from specimen reports. This resulted in a total of 1870 cases for analysis.

### Ethical consideration

No ethical approval was sought as the study did not include patient identifiable data.

## Results

A total of 2510 records were retrieved from the archives at the MakCHS Lab. Having excluded 640 records, eventually 1870 records were analyzed.

Females made up 97.3% of all the analyzed data. The female to male ratio for breast disease overall was 36:1.

Just over two thirds of the breast diseases diagnosed over the study period were benign (1271 cases, 68%), just under one third were malignant diseases (586 cases, 31.3%) and those precancerous (ductal and lobular carcinoma in situ) accounted for the remaining proportion (13 cases, 0.7%). The greater majority of the benign breast diseases were proliferative without atypia (825 cases, 65%), respectively followed by the non-proliferative group (434 cases, 34.1%) and those proliferative with atypia (12 cases, 0.9%).

The five most frequently diagnosed benign diseases overall were fibroadenoma (757 cases, 59.6%), fibrocystic breast disease (227 cases, 17.9%), sclerosing adenosis (57 cases, 4.5%), mastitis (49 cases, 3.9%) and gynaecomastia (18 cases, 1.4%). All these conditions were much more diagnosed in females than in males. The distribution of these benign diseases by sex is showed in Table 1.

**Table 1:** Gender distribution of the most commonly diagnosed benign breast diseases at the MakCHS Histopathology lab for the period 2005–2014

Benign breast disease	Females	Males	Total
Fibro adenoma	751	6	757
Fibrocystic breast disease	218	9	227
Sclerosing adenosis	54	3	57
Mastitis	48	1	49
Gynaecomastia	0	18	18
Other benign breast disease	161	2	163
Total	1232	39	1271

There were 586 breast cancers in total, mostly diagnosed in females. Of these, the most frequently diagnosed types were infiltrating ductal carcinoma (326 cases, 55.6%), invasive lobular carcinoma (59 cases, 10.1%), papillary carcinoma (4 cases, 0.7%) and medullary carcinoma (4 cases, 0.7%). Other histopathologically specified malignant diseases comprised less than 0.5%. Among the unspecified malignant diseases, 166 cases (28.3%) were concluded as adenocarcinoma but the cellular type was unspecified. Another 18 cases (3.1%) were concluded as only “breast malignancy” without details on cellular type or type of dysplasia. The female to male breast cancer ratio was 48:1.The distribution of these cancerous breast diseases by sex is showed in Table 2.

The article "Breast diseases histologically diagnosed at a tertiary facility in Uganda (2005–2014)" was published in 2018. Journal: BMC Cancer.

**Table 2:** Gender distribution of the most commonly diagnosed cancerous breast diseases at the MakCHS Histopathology Lab 2005–2014 by gender

Cancerous Breast disease	Females	Males	Total
Infiltrating Ductal Carcinoma	319	7	326
Invasive Lobular Carcinoma	59	0	59
Papillary Carcinoma	4	0	4
Medullary Carcinoma	4	0	4
Other cancerous breast disease	188	5	193
Total	574	12	586

Cancers overall showed a steady increase in the absolute numbers diagnosed per year over the study period whereas the benign diseases did not show any preferential pattern (Fig. 1). Nonetheless, the benign diseases remained higher than the malignant diseases throughout the study period as seen in Fig. 1.

**Fig. 1:** Overall trends in frequency of breast diseases diagnosed at the MakCHS Histopathology lab over the period 2005–2014

### Distribution of the breast diseases by age, ethnicity and region of patient origin

#### Age

The median age for breast disease overall was 26 years (IQR: 20–43) with the mean age being 33 years (standard deviation ±16.46).The age of males ranged between 12 and 82 years while that of the females ranged between 1 to 91 years old. The median ages for the most frequent benign and cancerous diseases by sex are shown in Table 3. Overall, breast cancers were diagnosed in females 16 years earlier than in males (median age of diagnosis being 48 and 64 years respectively).

**Table 3:** Median ages by gender for benign and cancerous breast diseases diagnosed at the MakCHS Histopathology lab 2005–2014

Breast pathology type	Breast disease diagnosed	Female	Male	Both sexes
Benign	Fibroadenoma	20	23	20
	Fibrocystic breast disease	23	43	23
	Sclerosing adenosis	25	63	27
	Mastitis	35	60	35
	Gynaecomastia	n/a	28	28
	All benign diseases	21	38	21
Cancer	Ductal carcinoma	48	52	49
	Lobular carcinoma	47	n/a	47
	Papillary carcinoma	43	0	43
	Medullary carcinoma	45	0	45
	Adenocarcinoma unspecified	49	67	50
	“Breast Malignancy”	50	65	50
	All cancers	48	64	49
All breast diseases		26	49	26

#### Regions

Uganda is divided into four major regions per the Uganda National Bureau of Statistics (UBOS) namely: Central, Western, Northern and Eastern. The MakCHS Lab is located in the country’s capital, Kampala which is in the Central region. The laboratory is no doubt the busiest histopathology laboratory in the country as it is the main public laboratory, serving the biggest hospital in the country and by far has the highest number of pathologists in the country. The central region was overrepresented contributing the biggest proportion of all breast diseases. The prevalence of breast cancer diagnosed from patients from Western region was comparatively higher than in other regions (Fig. 2).

The article "Breast diseases histologically diagnosed at a tertiary facility in Uganda (2005–2014)" was published in 2018. Journal: BMC Cancer.

**Fig. 2:** Graph showing regional distribution of breast diseases by type overall diagnosed at the MakCHS Histopathology Lab 2005–2014

## Discussion

This retrospective study was intended to give a general picture of the breast diagnoses made at a histopathology laboratory at a tertiary hospital in a Sub-Saharan African country. The study looked at breast records for ten years that is 2005–2014 inclusive.

2510 breast records were obtained for the entire period of study thus averaging about 250 records per year which seems to be small for such a population that has grown by several millions in a decade. Kampala alone where the laboratory is located has close to two million inhabitants. The low number maybe due to lower numbers of clinicians requesting for the service as evidenced by the referral hospital running only four breast clinics in a month, one per week. The burden of histopathology requests may also have been reduced by private laboratories within and around Kampala. However, the picture of sex distribution at this center does not differ from what is observed in many other studies and from the epidemiology of the disease. The greater occurrence of breast disease in females (97.1%) we observed concurs with the fact that male breast disease is generally lower than female breast disease [5].

Benign breast diseases were notably the commonest accounting for 68% of the diseases diagnosed in the ten years and this is similar globally [6]. It is known that benign breast disorders comprise the majority of presentations of breast disease at a breast clinic worldwide [6]. We did not however identify any of the patients earlier diagnosed with benign diseases later being diagnosed with cancers although it is known that some of the benign lesions may be pre-cancerous and that benign breast disease (BBD) generally poses a risk for breast cancer, which can develop later in either of the breasts [7]. We found a cancer prevalence of 31.2% of all the breast lesions diagnosed, this means that every 3 of 10 cases of breast diseases at the lab would end up as cancerous.

The article "Breast diseases histologically diagnosed at a tertiary facility in Uganda (2005–2014)" was published in 2018. Journal: BMC Cancer.

Most of the breast disease diagnosed in the country for the decade under study was benign, consistent with the fact that BBD is the most common form of breast disease worldwide [4].

Over the duration of study, fibroadenoma followed by fibrocystic breast disease were the most commonly diagnosed benign breast diseases overall. This was consistent with studies done in Uganda and Nigeria over the last 15 years [7–9]. This finding however was more evident in females since in males, gynaecomastia was the more predominant BBD being at least twice more common than either of fibroadenoma or FBC. Gynaecomastia is the most common male breast mass and because men generally lack lobular breast development, they are rarely diagnosed with fibroadenoma, FBC or other lobular breast condition [10].

We observed a consistent predominance in frequency of fibroadenoma over FBC throughout the decade which is different from findings in the western world and particularly the USA [11] where FBC has been documented to be more predominant than fibroadenoma. In parts of the Asia-pacific region [12], the two diseases have been noted to exchange predominance. Our findings may attest to the fact that the black race has been noted to have a racial predilection to fibroadenoma [13].

The most diagnosed breast cancer that we observed over the duration of study was infiltrating ductal carcinoma (326 cases, 55.6% of cancerous cases). This is consistent with findings in Africa, Europe and the world at large for the most frequently diagnosed breast cancer type [14, 15]. The fact that a considerable amount of records we retrieved were diagnosed or concluded only as either “adenocarcinoma” or “breast malignancy”, may explain why we observed less IDC compared to the documented 70–88% elsewhere [16–18]. More ancillary diagnostic techniques or better tissue harvest may be necessitated to counter this.

Nevertheless, we observed a pattern of increase in the frequency of diagnosis of breast cancer in the country, which was more profound in the last half of the study period. It has been noted as well that over the last 20 years, cancer incidence rates in older adults have been on the rise in Uganda, with breast cancer showing the largest increase (5%) in older adult females [19]. The increase we observed in occurrence of breast cancer by more than double from 21.2% in 2010 to 50.5% of all diagnosed breast disease in 2014 may nonetheless be reflective of a possible increase in the population’s utilization of laboratory diagnostic services. This may have been encouraged by a rise in specialized breast clinics especially in the private health sector, public health breast disease awareness campaigns, the several volunteer surgical camps within the districts and the increasing use of minimally invasive techniques like ultrasound guided core needle biopsy and breast disease screening using fine needle aspiration and cytology in both private and public health care settings. Furthermore, findings from breast cancer research projects running over the study period could potentially have been implemented in the communities pushing for better community health seeking behavior and clinical vigilance to improve early breast disease diagnosis and intervention resulting in increased breast clinic attendance and eventual increase breast cancer diagnosis rate represented by the observed positive trend in breast cancer diagnosis over the study duration.

The article "Breast diseases histologically diagnosed at a tertiary facility in Uganda (2005–2014)" was published in 2018. Journal: BMC Cancer.

Notwithstanding, the observed increase in breast cancer diagnosis may also be a clear reflection of increasing incidence of breast cancer in the country. It is of note that most majority of women in Uganda do not participate in breast cancer down-staging practices despite receiving breast cancer education, rather showing reference for breast health messaging from their health care providers [20]. This of course implies that where there is less health access across the country, most breast disease will be picked up in advanced stages, making referrals to the MakCHS Lab arrive as advanced breast disease. Moreover, the increasingly western lifestyle of the country’s populace cannot be overlooked as a modifiable role player in the observed trend in breast cancer incidence [21, 22].

The relatively low male breast cancer (MBC) rates we observed in Uganda over the study period (low male to female breast cancer ratio of 1:48), stand in agreement with the global picture where it has been observed that MBC, even though it has been noted to be increasing, comprises only about 0.8% of all the world’s diagnosed breast cancer [23]. Our findings showed a little less MBC in comparison with previous conclusions made about MBC rates in East Africa where male to female breast cancer ratios have been documented to range between 1:20–1:45 [24–26]. These observed rates though, are comparatively higher than those noted in Nigeria, West Africa 24 where the male to female breast cancer ratios approximated 1:70.

We further observed MBC in the country to occur just above a decade and a half (16 years) later in males than in females over the study period. Different parts of the world seem to show different comparative durations of onset for male versus female breast cancer. For instance, Nigeria [27] and Bangladesh [28] respectively show two decades and one decade for the median age of occurrence of MBC later than female breast cancer. All in all though, our findings and the findings of most of the studies worldwide agree to the occurrence of breast cancer later in males than in females. Most men may be seeking breast health care services later in life because of poor awareness about breast disease, stigma of male breast disease or other socio-cultural reasons [29].

The article "Breast diseases histologically diagnosed at a tertiary facility in Uganda (2005–2014)" was published in 2018. Journal: BMC Cancer.

Notwithstanding the above observations for breast cancer in the country, we observed breast disease in general, regardless of type, to largely occur at a young overall median age of 27 years. Our observed predominance of BBD in those under 35 years of age was similar to observations in the Asia-Pacific region, where for instance in China [30] and Japan [31], BBD has been increasingly diagnosed in the younger (less than 40 years) population. Much less breast disease was observed in individuals above 65 years of age. The modal age group we observed for a breast cancer diagnosis being 45 to 54 years means that most of the individuals diagnosed with breast cancer may have theoretically succumbed to the disease within or slightly above the observed modal age group. This alludes to the fact that Sub-Saharan Africa and Africa at large have been noted to have cancer survival rates that are generally poorer than for those individuals in higher income countries [32]. The average age range for a breast cancer diagnosis in Sub-Saharan Africa and the lower-income countries is 42 to 53 years [33]. The country’s low life expectancy (approximately 59 years) [34] may have an independent role leading to the observed discrepancy. Other reasons may also play a part in holding back the elderly from seeking services for breast health care and assessment such as; socio-cultural tendencies and related attitudes, cost of health care and stigma of breast disease.

Although each region of the country registered mostly benign breast diseases, the Western region showed the highest proportion of cancerous breast lesions for a single region (90 out of 203 cases, 44.3%). Most people from this region, notwithstanding the other regions of the country, may have accessed the MakCHS lab as a referral from a local regional health unit with breast disease that had already progressed from a pre-cancerous stage whereas those affected by benign breast disease may have been managed from local regional health units needless for referral. In some instances, individuals may have autonomously stayed home conscious of having breast disease, especially BBD, just like it has been observed in some other communities [35]. However, this does not eliminate the possibility of an environmental, dietary or genetic factor in the Western region of Uganda that allows modification of outcome of breast disease so that the likelihood of it progressing to a cancer is increased.

The article "Breast diseases histologically diagnosed at a tertiary facility in Uganda (2005–2014)" was published in 2018. Journal: BMC Cancer.

The Northern region had the lowest breast disease rates of any breast pathology type over the entire duration of study. This may be because of a comparatively less westernized dietary behavior or lifestyle in this region thus lowering an individual’s relative risk for having breast disease. The impact of the devastating war in the Northern region of Uganda, which fueled by the rebel Kony’s Lord’s Resistance Army for most of the period 1987 to the early 2000s resulted in massive loss of lives and gross retardation in the region’s health care delivery, service and referral systems, cannot be understated. These amongst other reasons may offer explanation for the observed breast disease rates in the Northern region. However, from this noted background, the region may benefit from multi-modal education efforts in radiological diagnosis of breast disease to augment early breast cancer detection using the comparatively less available but present radiologic modalities like breast ultrasound [36].

Overall however, the variations in regional distribution of breast disease may be reflective of the uneven distribution of breast disease diagnostic facilities or services throughout the country since arguably the greatest presence of these resources is found in the country’s Central region.

## Conclusions

The biggest proportion of breast disease diagnosed at the MakCHS Lab from 2005 to 2014 inclusive was in females. Most of this was BBD, the commonest being fibroadenoma. Breast cancer occurred up to 16 years later in males than in females. The commonest breast cancer in both males and females was invasive ductal carcinoma. There was an increase in both benign and malignant breast disease diagnosed over the study period. This increase in diagnosis was more rapid for malignant breast disease over the last half of the study period. The highest regional breast cancer proportion was from the Western region of the Country.

## Recommendations

There is need for more research into the picture of breast disease in the country, covering various demographic characteristics of the country’s population for all regions and informing about its incidence rates and prevalence and also the breast cancer risk estimate for benign breast disease.

## Abbreviations

BBD: Benign breast disease
FBC: Fibrocystic breast disease.
IDC: Invasive ductal carcinoma
IQR: Inter-quartile range
MakCHS Lab: Histopathology laboratory of the Department of Pathology of the Makerere University College of Health Sciences
MakCHS: Makerere University College of Health Sciences
MBC: Male breast cancer
UBOS: Uganda Bureau of Statistics
